The article "Using a Computer-Based Virtual Environment to Assess Social Cognition in Aging: An Exploratory Study of the REALSoCog Task" was published in 2022. Journal: Front Psychol.

# Using a Computer-Based Virtual Environment to Assess Social Cognition in Aging: An Exploratory Study of the REALSoCog Task

**DOI:** 10.3389/fpsyg.2022.882165

**Published:** 2022-05-17

**Authors:** Eva-Flore Msika, Nathalie Ehrlé, Alexandre Gaston-Bellegarde, Eric Orriols, Pascale Piolino, Pauline Narme

**Affiliations:** ^1^MC^2^Lab (UR 7536), Institut de Psychologie, Université Paris Cité, Paris, France; ^2^Service de Neurologie, CHRU Maison-Blanche, Reims, France

**Keywords:** social norms, emotional reactivity, empathy, theory of mind, moral cognition, social behavior, virtual reality

## Abstract

Although previous studies have suggested that some component processes of social cognition decline in normal aging, several methodological limitations can be pointed out. Traditional sociocognitive tasks assess processes separately and lack ecological validity. In the present study, the main aim was to propose an integrative social cognition assessment in normal aging using an original computer-based task developed in non-immersive virtual reality. Forty-five young adults (YA) and 50 older adults (OA) were asked to navigate in a simulated city environment and to judge several situations that they encountered. These situations investigated social norms by displaying control or (conventional/moral) transgressions. Following each situation, the participants were asked several questions in order to assess their ability to make moral judgments, affective and cognitive theory of mind, emotional reactivity and empathy, and the propensity to act in a socially appropriate or inappropriate way. The main results showed (i) a preserved ability to detect moral and conventional transgressions with advancing age; (ii) participants’ preserved cognitive ToM abilities; (iii) an age-related decline in affective ToM, that disappeared when the victim was a senior; (iv) preserved emotional reactivity and emotional empathy in normal aging; (v) an increase in inappropriate behavioral intentions in normal aging. Offering more naturalistic conditions, this new task is an interesting integrative measure of sociocognitive functioning to better reflect social behavior in daily living.

## Introduction

Since the 1970s, the cognitive revolution has led to an increasing interest in several functions in neuropsychology, particularly social cognition. The human being is studied through a social lens, as someone able to perceive and process social signals in order to behave appropriately during daily interpersonal relationships. More than 13,000 studies dealing with social cognition have been published during the last 5 years (PubMed). However, moral cognition and the knowledge of social conventions remain less studied than other well-known sociocognitive processes such as theory of mind (ToM) or empathy. Although morality can be understood as a unified concept from a functional point of view, it appears as a complex entity from a cognitive perspective (Greene, 2015), moral judgments being based on the integration of several inputs (e.g., emotions, others’ mental states, social knowledge, context, intentionality…) and underpinning adapted behavior (Mikhail, 2007). Thus, moral cognition might offer an interesting way to better understand how higher-order sociocognitive functions are integrated and/or interact with one another—another gap in the current literature on the neuropsychology of social cognition (Cassel et al., 2016; Etchepare and Prouteau, 2018).

The article "Using a Computer-Based Virtual Environment to Assess Social Cognition in Aging: An Exploratory Study of the REALSoCog Task" was published in 2022. Journal: Front Psychol.

Social cognition refers to a wide range of emotional and cognitive processes that enable humans to perceive and understand others’ emotions and mental states to adjust their own behavior (Shany-Ur and Rankin, 2011; Etchepare and Prouteau, 2018). A large distributed cerebral network involving prefrontal, temporal and insular structures is required for appropriate social interactions as it underpins accurate emotion recognition, ToM, empathy, and moral cognition (Kennedy and Adophs, 2012; Noonan et al., 2018). Emotion recognition involves perceptual capacities for decoding and making meaning out of emotional expressions using facial, prosodic or postural cues (McDonald, 2017). ToM refers to the ability to make inferences about others’ mental states in order to explain and predict their behavior (Premack and Woodruff, 1978; Conway and Bird, 2018). A distinction is usually made between cognitive and affective ToM (Brothers and Ring, 1992; Shamay-Tsoory and Aharon-Peretz, 2007). The former refers to the knowledge about others’ beliefs and/or intentions, whereas the latter corresponds to the understanding of others’ emotional states. Empathy, defined as the ability to share and understand another person’s feelings (Decety and Jackson, 2004), relies on two dissociable systems: the affective sharing of the pain and distress of others (i.e., emotional empathy) and the ability to adopt another’s psychological point of view (cognitive empathy; Shamay-Tsoory et al., 2009). Emotional empathy underlies empathic concern, defined as “other-oriented feelings of sympathy and concern for unfortunate others” (Davis, 1983, p. 114), which is particularly associated with a propensity to prosocial behavior. Cognitive empathy requires ToM processes but also the self-other distinction, top-down regulation processes and executive functions such as flexibility and inhibition (Preckel et al., 2018; Stietz et al., 2019). Finally, moral cognition corresponds to a set of capacities by which people learn, store and activate conventional and moral norms to make judgments and decisions about these norms (i.e., to decide whether an action is right or wrong; Haidt et al., 1993; Tasso et al., 2017; Voiklis and Malle, 2017). Conventional norms (e.g., eating with your hands) are mainly based on cultural rules, whereas moral norms (e.g., physically or emotionally hurting someone) appear more universal and involve emotional reactions (Hollos et al., 1986). Although both are judged as not permissible, moral transgressions (i.e., violation of a moral rule) are usually judged more severely than conventional transgressions (i.e., violation of a conventional rule; Blair, 1995; Nichols, 2002; Turiel, 2002). Moral judgment relies on the understanding of others’ mental states (i.e., judging the intentionality of action; inferring the victim’s emotional state), the semantic knowledge of norms but also on emotional abilities (Blair, 1995; Moll et al., 2005; Prinz, 2006; Young and Koenigs, 2007), for instance our level of empathic concern (Gleichgerrcht and Young, 2013). Thus, as predicted by Greene’s dual-process model (Greene, 2013), moral judgments are driven both by intuitive emotional responses and by conscious reasoning processes.

The article "Using a Computer-Based Virtual Environment to Assess Social Cognition in Aging: An Exploratory Study of the REALSoCog Task" was published in 2022. Journal: Front Psychol.

Social cognition is important for life satisfaction, social interactions and lower degrees of loneliness, especially in old age. However, previous studies have suggested that some component processes of social understanding may decline in normal aging. First, emotion recognition is classically described as being lower in older adults, especially when participants are asked to identify negative emotions (e.g., Ruffman et al., 2008; Birmingham et al., 2018; Visser, 2020). Considering ToM, although findings are equivocal (e.g., Happé et al., 1998; MacPherson et al., 2002; Wang and Su, 2013), most of the previous studies showed that increasing age results in decreased performance on ToM tasks, especially when assessing cognitive ToM (Duval et al., 2011; Henry et al., 2013; Bottiroli et al., 2016; Laillier et al., 2019). Thus, older adults show reduced levels of cognitive empathy (see Beadle and de la Vega, 2019 for a recent review). On the contrary, there is little evidence that emotional empathy decreases in aging. Previous findings rather suggest that emotional empathy is similar to or even higher in older than in younger adults, especially for empathic concern (Sze et al., 2012; Ze et al., 2014; Reiter et al., 2017; Beadle and de la Vega, 2019). Consistently, previous findings suggested that older adults might be more motivated than younger adults to help others (Sze et al., 2012; Rosi et al., 2019; Mayr and Freund, 2020). Overall, the processes underlying moral judgments seem to be impacted by aging. However, surprisingly—the issue of whether and how moral judgments and social norms might change in normal aging remains poorly explored (Moran et al., 2012; Baksh et al., 2018; Margoni et al., 2018). Moran et al. (2012) investigated whether aging was associated with difficulties in making an intent-based moral judgment. This kind of judgment is based on the agent’s intentions, blaming intentional harmful acts more than accidental ones. Unlike their younger counterparts, older adults relied less on intentions than on outcomes in their moral judgments (Moran et al., 2012). Margoni et al. (2018) replicated these findings and extended them by showing that (i) this age-related change was associated with a decline in ToM and (ii) no age-related change was observed for the moral evaluation of helpful actions. Furthermore, using a new task to assess different components of social cognition within the same test, Baksh et al. (2018) showed that increasing age was predictive of poorer performance on the interpersonal understanding of social norms (Baksh et al., 2018).

The article "Using a Computer-Based Virtual Environment to Assess Social Cognition in Aging: An Exploratory Study of the REALSoCog Task" was published in 2022. Journal: Front Psychol.

However, methodological limitations of traditional sociocognitive tasks might be pointed out. First, most of previous studies assessed social cognitive processes separately from one another, preventing an integrative assessment of social cognition. Few studies in the literature have investigated the different aspects of social cognition (Dziobek et al., 2008) by including conventional and moral judgments within the same task (Baksh et al., 2018). Second, the way the age-related decline of social cognition influences older adults’ intention to act/react has been poorly assessed, except for the link between empathy and prosocial behavior in some studies (e.g., Beadle et al., 2015). This point seems crucial to better understand the impairments of social behavior in the pathological framework. Finally, previous authors have pointed out the lack of ecological validity of sociocognitive tasks usually proposed (Isaacowitz and Stanley, 2011; Dziobek, 2012; Dawson and Marcotte, 2017; Sohlberg et al., 2019). In daily life situations, people are able to interpret others’ emotions and mental states as they dynamically evolve. Consistently, it appears that when using a dynamic presentation, emotion recognition is significantly higher (Lambrecht et al., 2012; Grainger et al., 2015) and cerebral activations underlying social cognition are stronger than when using photographs (Kilts et al., 2003; Trautmann et al., 2009). Also, in daily life experience, we rely not only on several key cues from the communicator (such as their voice, posture and bodily expressions), but also from contextual information (Achim et al., 2013; Duclos et al., 2018; Allain et al., 2020). Taking these limits into account, with more naturalistic conditions the technological possibilities offered by virtual reality (VR), even with non-immersive settings (i.e., Zhang et al., 2003; Cushman et al., 2008) or by serious games (Parsons and Courtney, 2001; Baldwin and Dandeneau, 2009; Kato and de Klerk, 2017), might be an interesting alternative to assess sociocognitive abilities. Indeed, immersive as well as non-immersive VR offers the opportunity to assess social cognition within an integrative context because of richer visual and contextual cues. Its playful properties provide a better participant involvement while allowing for the precise presentation and control of dynamic multi-sensory 3D stimulus environments (Rizzo et al., 2004). Previous research in clinical settings showed that non-immersive VR-based measures may be more sensitive in the detection and treatment of cognitive impairments than traditional methods (e.g., Allain et al., 2014; Foloppe et al., 2018; see also Liu et al., 2019 for a recent review). The main aim of the present study was to assess moral cognition and the different related components of social cognition in a integrative manner, in order to investigate (i) the presence of an age-related decline in the way participants detect and assess conventional and moral transgressions; (ii) the presence of an age-related decline in ToM and empathy; (iii) the intention to react toward the social situations encountered during the task. For this purpose, an original task was developed using non-immersive VR to assess social cognition in more naturalistic conditions. A secondary objective was to investigate relationships between moral cognition and other sociocognitive processes. Based on the previous findings, we expected an age-related decline in detecting and assessing conventional and moral transgressions and poorer performance in ToM. However, empathic concern and participants’ emotions following transgressions might be higher in older adults, associated with more intentions to react (e.g., to help others in need).

The article "Using a Computer-Based Virtual Environment to Assess Social Cognition in Aging: An Exploratory Study of the REALSoCog Task" was published in 2022. Journal: Front Psychol.

## Materials and Methods

### Participants

A total of 45 young adults (YA) and 50 healthy older adults (OA) were included. Participants were recruited from the surrounding community. They were all native French speakers. Using a quick health questionnaire, the absence of major neurological or psychiatric history was checked. Exclusion criteria were as follows: (i) a score above 8 obtained on the French Beck Depression Inventory-II (13-item version; Collet and Cottraux, 1986); and (ii) a score below the 5th percentile obtained on the Mini-Mental State French version (Kalafat et al., 2003) in OA. One OA participant was excluded based on the first criterion. All participants gave their written informed consent to participate in the study, which was conducted in compliance with the Helsinki Declaration. This study was reviewed and approved by the Comité d’Ethique de la Recherche de l’Université Paris Cité, n°IRB: 00012020-115.

We also screened whether participants misunderstood situations from the experimental sociocognitive task as suggested by a comprehension score below 90% (see below for a detailed description of the task). Based on this criterion, 4 OA participants were excluded. The characteristics of the remaining participants are summarized in Table 1.

**TABLE 1:** Participant characteristics.

	Young adults (*n* = 47)	Older adults (*n* = 45)	*p*
Age (years)	24.79 (4.61)	72.27 (6.50)	<0.001
Gender (Male/Female)	20/27	15/30	0.368
Education (years)	14.91 (2.83)	13.13 (3.25)	0.006
BDI-II (/39)	1.96 (2.51)	2.24 (2.06)	0.551
MMSE (/30)	−	28.53 (1.44)	−

*Data are expressed in mean (standard deviation). BDI-II, Beck Depression Inventory; MMSE, Mini-Mental State Examination.*

The two groups differed significantly in age, *t*_(1, 90)_ = 40.54, *p* < 0.001, and educational level *t*_(1, 90)_ = 2.81, *p* < 0.05. The gender distribution, *t*_(1, 90)_ = 0.91, *p* = 0.37, and the BDI-13 score, *t*_(1, 90)_ = 0.60, *p* = 0.55, did not differ significantly.

### The REALSoCog Task

The participants in the 2 groups were asked to carry out a non-immersive VR task, the REALSoCog task, developed by the Memory, Brain, and Cognition laboratory (MC^2^Lab, UR 7536) of the Institute of Psychology of Université Paris Cité. The environment and situations were built by two engineers of the MC^2^Lab, Alexandre Gaston-Bellegarde and Eric Orriols, using the Unity 3D and Mixamo Fuse tools for avatars, while the task was elaborated by Pauline Narme and Nathalie Ehrlé. The participants were asked “to navigate” in a virtual city in order to go to the train station, following a defined path indicated by yellow arrows. This paradigm was inspired from previous studies conducted in aging (Abichou et al., 2019, 2020). They were told to pay attention to several situations encountered during their navigation and were asked to judge them according to what most people would think about these situations.

A total of 27 situations were selected to assess the participants’ social cognitive processes (11 control/neutral situations and 16 experimental situations; cf. Figure 1). The experimental situations were specifically developed to investigate social norms by displaying conventional transgressions (e.g., a naked woman dancing in the street; *n* = 9) and moral transgressions (e.g., a child being robbed of money; *n* = 4). These situations were developed to elicit negative emotions and/or to show intentionally malicious behaviors. The three remaining experimental situations aimed at assessing (i) whether participants complied with a prohibited behavior (a policeman ordered them to turn away from a crime scene) and (ii) how participants would empathize with people in need (*n* = 2; e.g., an older woman carrying groceries falls down). Several other characters were also present in the virtual city in order to make the environment more realistic. However, questions were asked only when the participant encountered a control or an experimental situation.

The article "Using a Computer-Based Virtual Environment to Assess Social Cognition in Aging: An Exploratory Study of the REALSoCog Task" was published in 2022. Journal: Front Psychol.

**FIGURE 1:** Example of social situations encountered in the virtual environment: **(A)** Conventional transgression (a driver honking a woman in a wheelchair); **(B)** control situation (a man asking the participant the time).

Three questions were common to all the situations, regardless of type (see Table 2). First, to assess the capacity to **detect/reject transgression** (i.e., moral cognition), participants were asked whether the situation seemed appropriate or inappropriate (e.g., social norms questions in the Socials Norms Questionnaires; Kramer et al., 2014). When the participant judged the situation as inappropriate, they were asked to assess the **transgression severity** (i.e., moral cognition) using a 5-point Likert scale (from 1: slightly inappropriate to 5: completely inappropriate; Moral and conventional judgments task from the BCS; Ehrlé et al., 2011; adapted from Blair, 1995). Second, the participants were asked to explain what they had understood about the situation (**understanding score**). Third, to assess their intention to act, we asked the participants whether they would like to do something in each situation (**action propensity**) and to specify their intention. On the latter point, a qualitative scoring was made after data acquisition to judge whether the actions proposed were themselves appropriate or inappropriate (**rate of inappropriate behaviors**; e.g., physical or verbal behavior which is morally or conventionally transgressive; is inappropriate; is disproportionate considering the situation; is incoherent; is indicative of an adherence to the environment; etc.; Processing skills assessment question in the Assessment of Interpersonal Problem Solving Skills; Donahoe et al., 1990).

**TABLE 2:** Sociocognitive processes assessed during the REALSoCog task.

Measure	Question	Response
**Regardless of the kind of situation**		
Transgression detection	Does the situation seem appropriate or inappropriate?	Appropriate/Inappropriate
Transgression severity	(If inappropriate) How inappropriate does it seem?	1: Slightly, 5: Completely
Understanding	What did you understand about this situation?	Open-ended response
Action propensity Rate of inappropriate behaviors	Would you like to do something? (If yes) What would you like to do?	Yes/No Open-ended response
**For experimental situations**		
**Affective ToM**		
Accuracy Intensity	What do you think the person is feeling? How intensely do you think the person is experiencing the given emotion?	Open-ended response 1: Slightly, 5: Completely
**Cognitive ToM**		
Intentionality Valence	Is the behavior intentional? According to you, the intention is:	Yes/No 1: Very malicious, 5: Very benevolent
Emotional reactivity/emotional empathy*		
Intensity Valence	How concerned do you feel? The emotion you feel is:	1: Slightly, 5 Completely 1: Very negative, 5: Very positive

*The emotional reactivity scores were computed by calculating the mean across all experimental situations displaying a transgression, while the emotional empathy scores were computed by calculating the mean only across experimental situations displaying a transgression involving a victim and experimental situations developed to elicit empathy.

The article "Using a Computer-Based Virtual Environment to Assess Social Cognition in Aging: An Exploratory Study of the REALSoCog Task" was published in 2022. Journal: Front Psychol.

Additional questions were only administered when participants encountered an experimental situation (see Table 2). In experimental situations (i.e., featuring a transgression and/or construct to elicit empathy), (*n* = 11), participants were asked to say “what do you think this person is feeling?” as a measure of **affective ToM accuracy** (e.g., ToM question in the Awkward Moments Test; Heavey et al., 2000; affective ToM in the ESCoT; Baksh et al., 2018), and to rate the degree to which they thought the character was experiencing the given emotion (from 1: slightly to 5: completely). The latter question refers to the measure of **affective ToM intensity.** Some situations were related to an increased motivation in the elderly allowing a better identification with the character, as the victim of the situation was a senior. For these situations, we established a specific affective TOM score **(motivated affective ToM).**

When the experimental situation concerned a conventional or moral transgression that clearly displayed malicious behavior by a character toward the participant or another avatar (*n* = 6), participants were asked whether the behavior was intentional (yes or no; **intentionality cognitive ToM**; ToM question in the Awkward Moments Test; Heavey et al., 2000) and then to judge whether the intention was malicious or benevolent using a 5-point Likert scale (from 1: very malicious to 5; very benevolent; **valence cognitive ToM**). To capture the participants’ emotion, they were asked to rate how concerned they felt when looking at each experimental situation displaying a transgression (*n* = 13) using a 5-point Likert scale (from 1: not at all to 5: completely; **emotional reactivity**). This question also led to the computation of a specific score for experimental situations developed to elicit empathy and transgressions involving a victim (*n* = 6; **emotional empathy**). In both cases, participants were finally asked to specify the valence of their emotions when looking at each situation (from 1: very negative to 5: very positive; **emotional reactivity valence** and **emotional empathy valence**; empathic concern question in the Empathy for Pain Task; Baez et al., 2015).

The article "Using a Computer-Based Virtual Environment to Assess Social Cognition in Aging: An Exploratory Study of the REALSoCog Task" was published in 2022. Journal: Front Psychol.

Overall, through these questions, the REALsoCog task provided the assessment of several sociocognitive processes: the ability to make moral and conventional judgments, emotional empathy, affective and cognitive TOM and the propensity to act in a socially appropriate or inappropriate way.

### Procedure

Participants were tested individually in a quiet room. First, the inclusion criteria were checked. Then, sociocognitive abilities were assessed using the REALSoCog task. The virtual environment was displayed using on a computer screen (a laptop Acer Swift 3, 14 inches, screen definition 1,366 × 768—processor Intel Core i3 6100 U, RAM 4 Go, graphic card Intel HD Graphics 520). Participants navigated using the arrow keys on the computer keyboard. No VR headset was used. This choice was made considering the perspective to use the REALSoCog task in clinical settings. The control and experimental situations were encountered in a pseudo-randomized order, which was fixed across participants. Navigation in the REALSoCog task needed a familiarization phase, which was proposed to the participants using the same virtual environment, except that the social situations were removed. This familiarization phase lasted until the participant felt comfortable with the use of the keyboard keys. After completion of the REALSoCog task, participants filled out the two post-virtual navigation questionnaires (see below). The whole procedure lasted approximately an hour and a quarter.

### Post-virtual Navigation Assessment

After completion of the sociocognitive task, participants filled out two questionnaires. The first one was composed of 4 items extracted from the revised version of the Immersive Tendencies Questionnaire (ITQ; designed by the UQO Cyberpsychology Laboratory; Robillard et al., 2002; original version by Witmer and Singer, 1998). The 4 items chosen corresponded to the “emotion” factor (e.g., “Have you ever been scared by something happening on a TV show or in a movie?”). Participants responded using a 7-point scale (from “never” to “always”). The higher the score was, the higher the immersive tendencies (maximum score about 28). The second questionnaire was composed of 10 items corresponding to the “realism” and “auditory” factors of the Presence Questionnaire (PQ; designed by the UQO Cyberpsychology Laboratory; Robillard et al., 2002; original version by Witmer and Singer, 1998). Participants also responded using a 7-point scale (from “never” to “always”). The higher the score, the higher the feeling of presence in the virtual environment (maximum score about 70). Thus, this second questionnaire more specifically assessed the feeling of presence related to the navigation in our experimental sociocognitive task.

The article "Using a Computer-Based Virtual Environment to Assess Social Cognition in Aging: An Exploratory Study of the REALSoCog Task" was published in 2022. Journal: Front Psychol.

### Statistics

Correct detections or attributions were all expressed in mean percentage and standard error of the mean, while questions associated with a 5-point Likert scale were expressed in mean scores and standard error of the mean. ANOVAs with repeated measures were conducted on detection scores and action propensity with group (YA, OA) as a between-subjects factor and situation (control vs. experimental or moral transgressions vs. conventional transgressions) as a within-subjects factor. An ANCOVA was further conducted by introducing the understanding score and educational level as covariates. This analysis is reported only when the effect of at least one covariate is significant. One-way ANOVAs were conducted separately with group as a between-subjects factor for each of the scores assessing cognitive and affective ToM, emotional reactivity or emotional empathy, but also to compare groups on post-virtual navigation variables. In order to investigate the sociocognitive processes underlying participants’ judgments about moral and conventional transgressions, a Pearson correlation analysis was also conducted separately in each age group to highlight potential age-related changes. The SPSS software (version 18.0.3) was used for statistical analyses, with a significance threshold set at *p* ≤ 0.05. The JASP software was used to calculate the Omega squared effect size metric (Lakens, 2013).

## Results

### The REALSoCog Task

#### Transgression Detection

An ANOVA with repeated measures on detection scores (expressed as a percentage of correct answers) was conducted with group (YA, OA) as a between-subjects factor and situation type (control, experimental) as a within-subjects factor. It revealed a main effect of group [*F*_(1, 90)_ = 10.08; *p* = 0.002; ω^2^ = 0.05], due to the poorer performance in OA than in YA (see Table 3). However, the group x situation type interaction was significant [*F*_(1, 90)_ = 7.88; *p* = 0.006; ω^2^ = 0.04]. The one-way ANOVA that further investigated the effect of situation type in each group showed that OA had more difficulty in detecting control situations (tending to say that they were inappropriate) than YA [*F*_(1, 90)_ = 17.01; *p* < 0.001; ω^2^ = 0.15], while OA detected transgressions as well as YA [see Table 3; *F*_(1, 90)_ = 0.04; *p* = 0.84; ω^2^ < 0.001]. However, the understanding score, although very high in both groups (OA: 96.05% ± 0.36; YA: 98.78% ± 0.35), differed significantly between groups [*F*_(1, 90)_ = 30.01; *p* < 0.001; ω^2^ = 0.24] due to the poorer performance in OA. When this factor was introduced as a covariate in an ANCOVA, the group effect and the interaction disappeared [*F*_(1, 89)_ = 0.68; *p* = 0.41; ω^2^ < 0.001 and *F*_(1, 89)_ = 0.59; *p* = 0.44; ω^2^ < 0.001 respectively]. Therefore, it seems that the tendency of OA to judge control situations as inappropriate was mainly explained by a lower understanding of some situations.

The article "Using a Computer-Based Virtual Environment to Assess Social Cognition in Aging: An Exploratory Study of the REALSoCog Task" was published in 2022. Journal: Front Psychol.

**TABLE 3:** Performance on sociocognitive measures from the REALSoCog task in young and older adults.

Measure	Young adults	Older adults	*p*
**Transgression detection (%)**	90.25 (1.20)	84.82 (1.22)	0.002*
Control situations	91.67 (1.76)	81.30 (1.80)	< 0.001*
Experimental situations	88.83 (1.67)	88.33 (1.71)	0.84
*After controlling for understanding*	88.31 (1.18)	86.84 (1.21)	0.41
Control situations	88.04 (1.61)	85.09 (1.65)	0.23
Experimental situations	88.59 (1.81)	88.58 (1.86)	0.99
Moral transgressions	86.17 (2.63)	87.78 (2.69)	0.67
Conventional transgressions	91.49 (1.68)	88.89 (1.71)	0.28
**Transgression severity (/5)**	4.13 (0.08)	4.27 (0.09)	0.24
Moral transgressions	4.27 (0.09)	4.37 (0.10)	0.47
Conventional transgressions	3.99 (0.71)	4.09 (0.68)	0.19
**Action propensity (%)**	37.18 (1.62)	37.23 (1.58)	0.98
Control situations	22.63 (1.66)	23.63 (1.69)	0.67
Experimental situations	51.73 (2.11)	50.83 (2.16)	0.76
Moral transgressions	56.38 (3.46)	58.33 (3.53)	0.69
Conventional transgressions	42.32 (2.78)	40.25 (2.84)	0.60
**Inappropriate behaviors (%)**	5.99 (1.54)	12.72 (1.58)	0.003*
Control situations	4.79 (14.32)	13.89 (19.98)	**0.01**
Experimental situations	7.20 (1.50)	11.55 (1.53)	**0.04**
Moral transgressions	7.80 (2.52)	8.15 (2.57)	0.92
Conventional transgressions	7.72 (2.53)	13.71 (2.58)	0.10
**Affective ToM**			
Accuracy (%)	68.28 (2.15)	52.53 (2.2)	< 0.001*
Intensity (/5)	4.28 (0.06)	4.13 (0.06)	0.055 τ
**Cognitive ToM**			
Intentionality (%)	90.43 (2.08)	86 (2.13)	0.17
Valence (/5)	1.77 (0.06)	1.86 (0.06)	0.29
**Emotional reactivity**			
Intensity (/5)	3.01 (0.1)	3.09 (0.1)	0.57
Valence (/5)	2.08 (0.06)	2.16 (0.06)	0.33
**Emotional empathy**			
Intensity (/5)	3.77 (0.1)	3.92 (0.1)	0.29
Valence (/5)	1.86 (0.09)	2.05 (0.09)	0.12

Data are expressed in mean (standard error of the mean). *Significant intergroup comparison; τ, trend. Bold values are significant intergroup comparisons.

The article "Using a Computer-Based Virtual Environment to Assess Social Cognition in Aging: An Exploratory Study of the REALSoCog Task" was published in 2022. Journal: Front Psychol.

An ANOVA with repeated measures was also conducted on detection scores (expressed as a percentage of correct answers) with group (YA, OA) as a between-subjects factor and the kind of transgression (moral, conventional) as a within-subjects factor. No significant effects were found [main effect of group: *F*_(1, 90)_ = 0.043; *p* = 0.84; ω^2^ < 0.001; main effect of transgression: *F*_(1, 90)_ = 2.44; *p* = 0.12; ω^2^ = 0.007; group × transgression interaction: *F*_(1, 90)_ = 1.05; *p* = 0.31; ω^2^ < 0.001]. Thus, participants detected moral and conventional transgressions equally well (see Table 3).

#### Transgression Severity

An ANOVA with repeated measures was conducted on severity scores (expressed as the mean score about 5) with group (YA, OA) as a between-subjects factor and the kind of transgression (moral, conventional) as a within-subjects factor. The main effect of group was not significant [*F*_(1, 90)_ = 1.42; *p* = 0.24; ω^2^ = 0.002], suggesting that OA and YA assessed transgression severity in the same way (see Table 3). The main effect of transgression was significant [*F*_(1, 90)_ = 10.40; *p* = 0.002; ω^2^ = 0.03] due to higher severity scores attributed for moral transgressions (4.32 ± 0.07) compared to conventional transgressions (4.09 ± 0.07). No group x transgression interaction was found [*F*_(1, 90)_ = 0.38; *p* = 0.54; ω^2^ < 0.001]. In other words, moral and conventional transgressions were judged by OA as severely as by YA, while moral transgressions were considered slightly more serious than conventional transgressions in both groups.

#### Theory of Mind

One-way ANOVAs were conducted separately on each ToM score with group (YA, OA) as a between-subjects factor. Considering affective ToM, analyses showed (i) a significant group effect on affective ToM accuracy [*F*_(1, 90)_ = 26.16; *p* < 0.001; ω^2^ = 0.22], due to a better performance in YA (68.28% ± 2.15) than in OA (52.53% ± 2.2); (ii) a trend to a group effect on affective ToM intensity of a medium effect size [*F*_(1, 90)_ = 3.77; *p* = 0.055; ω^2^ = 0.03] with a lower intensity judgment in OA (4.13 ± 0.06) than in YA (4.28 ± 0.06). Interestingly, the group effect on affective ToM accuracy disappeared when only situations involving a senior were considered [motivated affective ToM; *F*_(1, 90)_ = 2.43; *p* = 0.12; ω^2^ = 0.01]. Considering cognitive ToM, the group effect was not significant on intentionality cognitive ToM [YA: 90.43% ± 2.08; OA: 86% ± 2.13; *F*_(1, 90)_ = 1.92; *p* = 0.17; ω^2^ = 0.01] or valence cognitive ToM [YA: 1.77 ± 0.06; OA: 1.86 ± 0.06; *F*_(1, 90)_ = 1.14; *p* = 0.29; ω^2^ = 0.002].

The article "Using a Computer-Based Virtual Environment to Assess Social Cognition in Aging: An Exploratory Study of the REALSoCog Task" was published in 2022. Journal: Front Psychol.

#### Emotional Reactivity and Empathy

One-way ANOVAs were conducted separately on each emotional score with group (YA, OA) as a between-subjects factor. When looking at experimental situations displaying a transgression, the mean emotional reactivity scores from OA (3.09 ± 0.1) and YA (3.01 ± 0.1) were similar [*F*_(1, 90)_ = 0.33; *p* = 0.57; ω^2^ < 0.001]. Their mean emotional reactivity valence did not differ significantly [*F*_(1, 90)_ = 0.97; *p* = 0.33; ω^2^ < 0.001] but was more negative in OA (2.16 ± 0.06) than in YA (2.08 ± 0.06). When looking at empathic situations and transgressions involving a victim, the mean emotional empathy scores of OA (3.92 ± 0.1) and YA (3.77 ± 0.1) did not differ significantly [*F*_(1, 90)_ = 1.13; *p* = 0.29; ω^2^ < 0.001]. The findings were similar for mean emotional empathy valence [*F*_(1, 90)_ = 2.51; *p* = 0.12; ω^2^ = 0.02], but with slightly more negative scores in OA (2.05 ± 0.09) than in YA (1.86 ± 0.09).

#### Action Propensity

An ANOVA with repeated measures was conducted on action propensity (expressed as a percentage) with group (YA, OA) as a between-subjects factor and situation (control, experimental) as a within-subjects factor. The main effect of group was not significant [*F*_(1, 90)_ < 0.001; *p* = 0.98; ω^2^ < 0.001], suggesting that OA proposed to react to the situation as often as the YA did (see Table 3). A main effect of situation was found [*F*_(1, 90)_ = 356.03; *p* < 0.001; ω^2^ = 0.54], due to a higher action propensity in experimental situations (51.28% ± 1.51) than in control situations (23.13% ± 1.19). The group × situation interaction was not significant [*F*_(1, 90)_ = 0.41; *p* = 0.53; ω^2^ < 0.001]. To further investigate the action propensity toward experimental situations, an ANOVA with repeated measures was conducted on action propensity (expressed as a percentage) with group (YA, OA) as a between-subjects factor and transgression (moral, conventional) as a within-subjects factor. The main effect of group was not significant [*F*_(1, 90)_ < 0.001; *p* = 0.98; ω^2^ < 0.001], suggesting that OA proposed to react to the experimental situations as often as the YA did (respectively: 49.29% ± 2.63 and 49.35% ± 2.57). A main effect of transgression was found [*F*_(1, 90)_ = 38.99; *p* < 0.001; ω^2^ = 0.12], due to the higher proportion of actions proposed toward moral (57.36% ± 2.47) than conventional transgressions (41.28% ± 1.98). The group x transgression interaction was not significant [*F*_(1, 90)_ = 0.61; *p* = 0.44; ω^2^ < 0.001], suggesting that both groups reacted more frequently when considering moral rather than conventional transgressions.

The article "Using a Computer-Based Virtual Environment to Assess Social Cognition in Aging: An Exploratory Study of the REALSoCog Task" was published in 2022. Journal: Front Psychol.

We were also interested in the nature of the actions proposed by the participants, especially if these actions were assessed as inappropriate by the experimenters. An ANOVA with repeated measures was conducted on the rate of inappropriate behaviors (expressed as a percentage) with group (YA, OA) as a between-subjects factor and situation (control, experimental) as a within-subjects factor. The effect of situation and the group × situation interaction were not significant [*F*_(1, 90)_ < 0.001; *p* = 0.98; ω^2^ < 0.001; *F*_(1, 90)_ = 1.43; *p* = 0.24; ω^2^ = 0.002]. The main effect of group was the only significant effect but with a small effect size [*F*_(1, 90)_ = 9.29; *p* = 0.003; ω^2^ = 0.04], due to a higher proportion of inappropriate actions proposed by OA in comparison with YA (see Table 3). Finally, we checked the ANOVA with repeated measures on the rate of inappropriate behaviors (expressed as a percentage) with group (YA, OA) as a between-subjects factor and transgression (moral, conventional) as a within-subjects factor. No effect was significant [group: *F*_(1, 90)_ = 1.41; *p* = 0.24; ω^2^ = 0.002; transgression: *F*_(1, 90)_ = 1.28; *p* = 0.26; ω^2^ = 0.001; group × transgression: *F*_(1, 90)_ = 1.36; *p* = 0.25; ω^2^ = 0.002].

### Correlation and Regression Analyses

A correlation analysis was first conducted in each age group in order to investigate the sociocognitive processes underlying participants’ judgments about moral and conventional transgressions (detection accuracy and transgression severity; see Table 4). Subsequently a linear regression analysis was conducted for each relevant dependent variable by introducing significantly correlated measures as predictive variables.

**TABLE 4:** Correlations (Bravais-Pearson correlation coefficient) between transgression detection/severity and sociocognitive processes assessed during the REALSoCog task in young (YA) and older adults (OA).

	Emotional empathy	Emotional empathy valence	Emotional reactivity	Emotional reactivity valence	Affective ToM accuracy	Affective ToM intensity	Intentionality cognitive ToM	Valence cognitive ToM
***In YA***								
Moral transgressions								
Detection	0.27	–0.22	0.29*	−0.30*	0.18	0.18	–0.22	–0.26
Severity	0.24	–0.01	0.26	–0.25	0.18	0.41**	0.11	–0.27
Conventional transgressions								
Detection	0.45***	–0.22	0.43**	−0.42**	0.13	0.23	0.01	–0.16
Severity	0.43**	–0.06	0.60***	−0.48***	0.21	0.65***	0.08	–0.23
***In OA***								
Moral transgressions								
Detection	0.11	–0.13	–0.002	–0.12	–0.25	–0.09	–0.11	–0.09
Severity	0.25	–0.24	0.15	−0.32*	0.25	0.29	0.13	−0.40**
Conventional transgressions								
Detection	0.21	–0.04	–0.03	–0.24	–0.03	0.21	0.04	–0.19
Severity	0.05	0.13	0.28	–0.16	–0.08	0.31*	0.14	–0.02

*ToM, theory of mind.*

*p < 0.05; **p < 0.01; ***p < 0.001.

The article "Using a Computer-Based Virtual Environment to Assess Social Cognition in Aging: An Exploratory Study of the REALSoCog Task" was published in 2022. Journal: Front Psychol.

*Significant intergroup comparisons are indicated in bold.*

In young adults, their identification of moral transgressions was correlated with their emotional reactivity (*r* = 0.29; *p* < 0.05) and their emotional reactivity valence (*r* = −0.30; *p* < 0.05). The higher the emotional reactivity and the more negative the emotional reactivity valence when looking at experimental situations, the higher their ability to detect moral transgression. However, the linear regression analysis revealed no significant predictive factors (both *p* > 0.2). Their judgments of transgression severity were correlated with the intensity of others’ emotions (affective ToM intensity, *r* = 0.41; *p* = 0.004). The affective ToM intensity (β = 0.41; *p* = 0.004) statistically predicted judgments of moral transgression severity [*F*_(1, 45)_ = 9.2; *p* = 0.004; *R*^2^ = 0.17]. Considering the identification of conventional transgressions, it was correlated in YA with their emotional reactivity (*r* = 0.43; *p* < 0.05), their emotional reactivity valence (*r* = −0.42; *p* = 0.003), and their emotional empathy (*r* = 0.45; *p* = 0.001). However, the linear regression analysis revealed no significant predictive factors (all *p* > 0.1). Young adults’ judgments of the transgression severity were correlated with emotional reactivity (*r* = 0.60; *p* < 0.001), emotional reactivity valence (*r* = −0.48; *p* < 0.001), emotional empathy (*r* = 0.43; *p* = 0.003) and the intensity of others’ emotions (affective ToM intensity, *r* = 0.65; *p* < 0.001). The model statistically predicted judgments of conventional transgression severity [*F*_(4, 42)_ = 12.6; *p* < 0.001; *R*^2^ = 0.55]. Out of four, three variables added significantly to the prediction (emotional reactivity: β = 0.49; *p* = 0.004; emotional empathy: β = −0.39; *p* = 0.03; affective ToM intensity: β = 0.59; *p* = 0.001). Overall, it appears that young adults based their moral and conventional judgments of severity on their own emotions and those they may attribute to others.

In older adults, no significant correlation was found between their identification of moral or conventional transgressions and sociocognitive processes. However, their judgments of the severity for moral transgressions were correlated with their emotional reactivity valence (*r* = −0.32; *p* = 0.03) and the valence cognitive ToM (*r* = −0.40; *p* = 0.006). The more negative their emotional reactivity valence when looking at experimental situations and the more malicious the intention, the higher their judgment of moral transgression severity. The model statistically predicted judgments of moral transgression severity [*F*_(2, 42)_ = 5; *p* = 0.01; *R*^2^ = 0.19]. Out of two variables, the valence cognitive ToM only added significantly to the prediction (β = −0.33; *p* = 0.04). Older adults’ judgments of the severity for conventional transgressions were only correlated with the intensity of others’ emotions (affective ToM intensity, *r* = 0.31; *p* = 0.04). The affective ToM intensity (β = 0.31; *p* = 0.04) statistically predicted judgments of conventional transgression severity [*F*_(1, 43)_ = 4.6; *p* = 0.04; *R*^2^ = 0.10]. Overall, it seems that older adults (i) based their detection of transgression on other processes than those assessed in the REALSoCog task; (ii) judged the severity of moral transgressions based on the intentionality attributed to others’ behaviors, while the severity of conventional transgressions might depend on the emotion intensity attributed to others.

The article "Using a Computer-Based Virtual Environment to Assess Social Cognition in Aging: An Exploratory Study of the REALSoCog Task" was published in 2022. Journal: Front Psychol.

Considering the theoretical proximity in the moral psychology field between ToM and empathy (Dvash and Shamay-Tsoory, 2014; Zucchelli and Ugazio, 2019), an additional correlation analysis was conducted to investigate whether empathy and ToM scores (respectively, emotional empathy intensity/valence, affective ToM accuracy/intensity and cognitive ToM accuracy/intensity) were highly related in the present task. Taking into account the whole sample, results showed that when looking at experimental situations developed to elicit empathy and transgressions involving a victim (i) more participants thought the character was experiencing an emotion (affective ToM intensity), more they felt concerned (emotional empathy intensity; *r* = 0.64; *p* < 0.001) and more negative was their emotion (emotional empathy valence; *r* = 0.3; *p* = 0.004); (ii) more malicious was judged the transgression intention (cognitive ToM valence), more negative was the participants’ emotion (*r* = −0.37; *p* < 0.001). No other correlation was significant (all *p* > 0.1).

### Post-virtual Navigation Assessment

Between-group comparisons on the Emotion ITQ score showed that YA and OA differed significantly in their immersive tendencies in everyday life [*F*_(1, 90)_ = 18.4, *p* < 0.001; ω^2^ = 0.16]. Older adults were less likely to become immersed in a virtual environment (11.84 ± 0.77) than YA (16.49 ± 0.76; maximum score about 18). However, as shown by their scores on items from the PQ questionnaire (maximum score about 70), OA felt as immersed as YA during the REALSoCog task [respectively, 45.13 ± 1.39 and 42.87 ± 1.38; *F*_(1, 90)_ = 1.36, *p* = 0.25; ω^2^ = 0.004]. Thus, the previous reported differences in sociocognitive scores could not be better explained by differences in their feeling of presence.

The article "Using a Computer-Based Virtual Environment to Assess Social Cognition in Aging: An Exploratory Study of the REALSoCog Task" was published in 2022. Journal: Front Psychol.

### Control for the Educational Level Effect

To ensure that the educational level did not explain the OAs’ results pattern, additional control was conducted by dividing the OA group according to their educational level. Based on the median score, 23 OA with a level equal or below 13 years (10.4 ± 1.7) were compared to 22 OA with a higher level by using *t*-tests for independent groups (16 ± 1.6). Results showed that the educational level only impacts significantly the detection of control situations [*t*(43) = −2.5; *p* = 0.02] and the propensity to act when looking at moral transgressions [*t*(43) = 2; *p* = 0.05] but not to the one to behave inappropriately [*t*(43) = 0.5; *p* > 0.6]. In these cases, OA with a lower educational level obtained lower performances than those with higher educational level (respectively, for the detection of control situations: 76.4 ± 13.7 vs. 86.4 ± 12.5: for the propensity to act when looking at moral transgressions: 66.3 ± 27.8 vs. 50 ± 26.7).

## Discussion

The present study was designed to assess different sociocognitive processes within the same task, in order to investigate a potential decline in detecting and judging moral and conventional transgressions as well as potential age-related changes in ToM and/or empathy. We also wanted to assess participants’ intention to react toward social situations. To investigate these issues, a new sociocognitive task was developed and proposed to young and older adults. The originality of this computer-based virtual task (REALSoCog) is that it aimed to assess several sociocognitive processes within the same task, in more naturalistic conditions. A secondary purpose was to investigate relationships between moral cognition and other sociocognitive processes.

Our results first showed a preserved ability to accurately detect moral and conventional transgressions with advancing age. This result is somewhat debatable, however, as OA tended to detect transgressions when there are none (i.e., in control situations). Cohort and generational factors may play a role, as YA were more permissive toward behaviors that were once more reprehensible (e.g., wearing a mini skirt). However, this age-related over-rating of transgressions existed only in lower educated OA and disappeared when the lower understanding of some social situations among OA was considered. Consistently, the transgression severity judgments seem to be similar in both groups with a distinction between moral and conventional norms, moral transgressions being more severely judged than conventional ones (Turiel, 1983; Ehrlé et al., 2011). Taken together, these results suggest—contrary to our expectations—the absence of age-related decline in the way participants detect and assess moral and conventional transgressions (see Moran et al., 2012; Margoni et al., 2018 for convergent results). Older adults’ judgments might be based on the agent’s intentionality rather than on outcomes, as in YA. In both groups, our results suggest a regulation of participants’ judgments (especially in terms of their assessment of the seriousness of transgressions). A thorough examination of why they judged behavior as a transgression by exploring participants’ oral justifications supporting their moral reasoning could help to specify age-related changes.

The article "Using a Computer-Based Virtual Environment to Assess Social Cognition in Aging: An Exploratory Study of the REALSoCog Task" was published in 2022. Journal: Front Psychol.

Second, the present results showed differential effects of normal aging on ToM depending on the component considered. Cognitive ToM appears to be preserved in OA while age-related decline concerns affective ToM here (see Henry et al., 2013 for a meta-analysis). REALSoCog proposes a first-order cognitive ToM assessment, which is well preserved in aging (McKinnon and Moscovitch, 2007; Duval et al., 2011) because less cognitively costly (Maylor et al., 2002) than the second-order cognitive TOM. Consistently with previous studies, OA performance decreases when it comes to inferring affective mental states (Slessor et al., 2007; Bailey and Henry, 2008; Duval et al., 2011; Fischer et al., 2017; Fernandes et al., 2019). The executive cost, especially inhibition capacities that are altered with age, is likely to contribute to these difficulties (Bailey and Henry, 2008; Duval et al., 2011; Wang and Su, 2013; Fischer et al., 2017). The relative preservation of cognitive ToM abilities in our cohort of OA could explain why they did not show any decline in moral/conventional judgments. Indeed, Moran et al. (2012) proposed that an age-related decline in cognitive ToM disturbs the way older participants infer the agent’s intentionality during moral reasoning. On the other hand, it is interesting that the difficulties in affective ToM disappeared when the victim was a senior. In other words, when faced with situations that favor taking the other character’s perspective and facilitate identification, the mentalization abilities of OA seem increased (see Sze et al., 2012 for convergent conclusions regarding empathy).

The article "Using a Computer-Based Virtual Environment to Assess Social Cognition in Aging: An Exploratory Study of the REALSoCog Task" was published in 2022. Journal: Front Psychol.

Third, our results showed that emotional reactivity and emotional empathy are preserved in normal aging (see also, Beadle et al., 2015; Reiter et al., 2017; Bailey et al., 2020). Although these results do not support the hypothesis of higher emotional empathy with advancing age, they might contribute to the current debate in the literature as to whether empathy levels increase in the elderly or not (Sze et al., 2012; Beadle et al., 2015; Wieck and Kunzmann, 2015; Bailey et al., 2020). REALSoCog offers a state assessment of emotional empathy, corresponding to a punctual and contextual emotional reaction provoked by observing the suffering of others. Unlike most tools used to assess this component in previous studies, it enables an objective measure that avoids the limitations associated with traditional self-evaluations, which may be biased due to social desirability (Beadle and de la Vega, 2019).

Finally, our results suggest that OA did not increase their intentions to act when looking at moral and social transgressions. However, in contrast with previous studies showing that OA are more likely to be involved in prosocial behaviors (Sze et al., 2012; Rosi et al., 2019; Mayr and Freund, 2020), this result is consistent with the observation of a similar emotional empathy and emotional reactivity to that of YA. Indeed, these components modulate social behavior: the personal involvement felt by a subject when judging a transgression predicts their propensity to share their disapproval (Brauer and Chekroun, 2005; Helweg-Larsen and LoMonaco, 2008). This is consistent with the finding of a greater action propensity for moral transgressions compared to conventional transgressions in both groups, the former being deemed more serious than the latter (Turiel, 1983), and therefore more likely to involve subjects emotionally. It should be highlighted that REALSoCog demonstrated a significant—but small—increase in inappropriate behavioral intentions in OA. These results might argue in favor of the sensitivity of the tool proposed, since inappropriate social behavior is not systematically detected by peers (Henry et al., 2009).

Considering our secondary goal of investigating relationships between moral cognition and other sociocognitive processes, we found slightly different patterns in YA and OA. Our regression analyses showed that, consistent with previous studies (Voiklis and Malle, 2017), YA’s moral/conventional judgments seem to rely on the agent’s intentions and on an analysis of mental states (especially in terms of their assessment of the intensity of others’ emotions), but also on the analysis of their own mental state (in terms of emotions they feel). This result suggests a double influence of the “social brain” and the “emotional brain” (Young and Dungan, 2012) in moral/conventional judgments (Greene et al., 2001; Nichols, 2002; Moll et al., 2008; Tasso et al., 2017; Bretz and Sun, 2018). In contrast, OA’s moral/conventional judgments did not rely on their own emotions but only on the analysis of others’ mental states (in terms of the others’ intentionality and the intensity of others’ emotions). Overall, this exploratory study suggests that REALSoCog could be an interesting task to assess sociocognitive processes in normal aging. This task seems to provide an objective assessment of some social cognitive aspects (especially emotional empathy and social behaviors), which are often only assessed based on subjective tools. Although the sociocognitive functioning of OA is marked by considerable inter-individual heterogeneity, requiring caution in generalizing the results of the present study, it has also to be underlined that the nature of the task itself may explain some discrepancies with results reported in the literature. Offering more naturalistic conditions, this computer-based virtual task may have reduced the involvement of other non-social cognitive functions that can interfere with the social cognitive functioning in OA, thus contributing to the finding that fewer age-related changes were revealed using the REALSoCog task in comparison with the classical tasks used in the literature. Although the acceptance or relevance of non-immersive VR could be questioned in the elderly due to a reduced exposure to this kind of technology in comparison with YA, it has to be underlined that our results cannot be explained by group differences in their feeling of immersion in the virtual environment, since comparable judgments were observed. Finally, the integrative measure of sociocognitive functioning may offer possibilities to investigate and better understand relationships between moral cognition and other sociocognitive processes such as theory of mind and empathy.

The article "Using a Computer-Based Virtual Environment to Assess Social Cognition in Aging: An Exploratory Study of the REALSoCog Task" was published in 2022. Journal: Front Psychol.

Nevertheless, methodological limitations need to be discussed. First, our experimental design did not allow to directly test the added value of the use of a virtual environment in comparison with classical tasks. Even whether the REALSoCog task is hypothesized to be more naturalistic offering a more ecologically valid assessment, we did not compare OAs’ performances on this task vs. on traditional tasks. Future studies are required to further investigate this issue to confirm the validity of the REALSoCog task. Second, although slightly lower than in the YA, the OA’s educational level was quite high in the present study. This may have compensated for age-related decline. However, when contrasting OAs’ performances according to their educational level, it appears that the pattern of lower educated OA was quite similar to the one observed in higher educated ones on moral cognition, ToM, empathy and declarative intentions of social behaviors. It should also be noted that an intergenerational comparison implies demographic and ideological pluralism, which can influence participants’ normative theory with changes in conventional norms over time (Turiel, 1983). Furthermore, the test is long and can lead to fatigue and/or disinvestment by the participants. Some situations were also associated with ambiguous interpretations as suggested by the corresponding understanding score. In a future study, item analysis will contribute to selecting the most reliable situations for a shorter version of the task. Basic perceptual differences between YA and OA might have contributed to explain some of the age-related decline observed. Such abilities should have been controlled. This is also the case for potential cybersickness symptoms (Kourtesis et al., 2020) or differences in the familiarity with using computer devices (Zygouris and Tsolaki, 2015), where both may have affected performances. Considering the former, it has to be underlined that cybersickness symptoms are mainly associated with immersive VR (Plechatá et al., 2019). Although we cannot totally rule out the presence of such symptoms in our results, it should be noted that in case of non-immersive VR, these symptoms appear after long time exposure (Tazawa and Okada, 2001) while this is not the case with the REALSoCog task. For the latter point, although OA might be less familiar with using computers, all our participants were trained with the simulated city environment for as long as they needed before the experimental task.

This integrative social cognition task will offer both theoretical and clinical perspectives. From a theoretical point of view, it may provide an interesting way to better understand how higher-order sociocognitive functions are integrated and/or interact with each other, which is currently a gap in the literature on the neuropsychology of social cognition (Cassel et al., 2016; Achim et al., 2020). From a clinical point of view, despite its interest for both diagnostic and rehabilitation purposes, the neuropsychological assessment of social cognition remains underexamined in clinical practice mainly due to a lack of reliable tools (Kelly et al., 2017). Thus, future studies should investigate the validity and the potential value of the REALSoCog task in clinical neuropsychology, as well as clarify the sociocognitive processes interdependency. A more immersive and interactive version of this task may also be of interest.

The article "Using a Computer-Based Virtual Environment to Assess Social Cognition in Aging: An Exploratory Study of the REALSoCog Task" was published in 2022. Journal: Front Psychol.

## Data Availability Statement

The raw data supporting the conclusions of this article will be made available by the authors, without undue reservation.

## Ethics Statement

The studies involving human participants were reviewed and approved by the Comité d’Ethique de la Recherche de l’Université Paris Cité, N°IRB: 00012020-115. The patients/participants provided their written informed consent to participate in this study.

## Author Contributions

PN, NE, and PP contributed to conception of the study. AG-B and EO contributed to design of the virtual environment and technical assistance. E-FM organized data collection, performed the statistical analysis, and wrote the first draft of the manuscript. PN wrote sections of the manuscript. All authors contributed to manuscript revision, read and approved and approved the submitted version.

## Conflict of Interest

The authors declare that the research was conducted in the absence of any commercial or financial relationships that could be construed as a potential conflict of interest.

## Publisher’s Note

All claims expressed in this article are solely those of the authors and do not necessarily represent those of their affiliated organizations, or those of the publisher, the editors and the reviewers. Any product that may be evaluated in this article, or claim that may be made by its manufacturer, is not guaranteed or endorsed by the publisher.
